The article "Adenosine and inosine exert cytoprotective effects in an in vitro model of liver ischemia-reperfusion injury" was published in 2012. Journal: Int J Mol Med.

# Adenosine and inosine exert cytoprotective effects in an *in vitro* model of liver ischemia-reperfusion injury

**DOI:** 10.3892/ijmm.2012.1203

**Published:** 2012-12-04

**Authors:** KATALIN MÓDIS, DOMOKOS GERŐ, RITA STANGL, OLIVÉR ROSERO, ATTILA SZIJÁRTÓ, GÁBOR LOTZ, PETRA MOHÁCSIK, PETRA SZOLECZKY, CIRO COLETTA, CSABA SZABÓ

**Affiliations:** 1 Department of Anesthesiology, University of Texas Medical Branch, Galveston, TX 77555, USA;; 2 CellScreen Applied Research Center, Semmelweis University Medical School, Budapest, Hungary; 3 1st Department of Surgery, Semmelweis University Medical School, Budapest, Hungary; 4 2nd Department of Pathology, Semmelweis University Medical School, Budapest, Hungary

**Keywords:** adenosine, inosine, cytoprotection, liver, ischemia-reperfusion, hepatocytes

## Abstract

Liver ischemia represents a common clinical problem. In the present study, using an *in vitro* model of hepatic ischemia-reperfusion injury, we evaluated the potential cytoprotective effect of the purine metabolites, such as adenosine and inosine, and studied the mode of their pharmacological actions. The human hepatocellular carcinoma-derived cell line HepG2 was subjected to combined oxygen-glucose deprivation (COGD; 0-14-24 h), followed by re-oxygenation (0-4-24 h). Adenosine or inosine (300–1,000 *μ*M) were applied in pretreatment. Cell viability and cytotoxicity were measured by the 3-(4,5-dimethyl-2-thiazolyl)-2,5-diphenyl-2H-tetrazolium bromide and lactate dehydrogenase methods, respectively. The results showed that both adenosine and inosine exerted cytoprotective effects, and these effects were not related to receptor-mediated actions, since they were not prevented by selective adenosine receptor antagonists. On the other hand, the adenosine deaminase inhibitor erythro-9-(2-hydroxy-3-nonyl) adenine hydrochloride (EHNA, 10 *μ*M) markedly and almost fully reversed the protective effect of adenosine during COGD, while it did not influence the cytoprotective effect of inosine in the same assay conditions. These results suggest that the cytoprotective effects are related to intracellular actions, and, in the case of adenosine also involve intracellular conversion to inosine. The likely interpretation of these findings is that inosine serves as an alternative source of energy to produce ATP during hypoxic conditions. The protective effects are also partially dependent on adenosine kinase, as the inhibitor 4-amino-5-(3-bromophenyl)-7-(6-morpholino-pyridin-3-yl)pyrido[2,3-d]pyrimidine, 2HCl (ABT 702, 30 *μ*M) significantly reversed the protective effect of both adenosine and inosine during hypoxia and re-oxygenation. Collectively, the current results support the view that during hypoxia, adenosine and inosine exert cytoprotective effects via receptor-independent, intracellular modes of action, which, in part, depend on the restoration of cellular bioenergetics. The present study supports the view that testing of inosine for protection against various forms of warm and cold liver ischemia is relevant.

The article "Adenosine and inosine exert cytoprotective effects in an in vitro model of liver ischemia-reperfusion injury" was published in 2012. Journal: Int J Mol Med.

## Introduction

Liver ischemia-reperfusion is a common problem in many clinical conditions such as liver transplantation, hepatic failure after shock, and liver surgery. Liver reperfusion injury not only causes liver dysfunction, but also frequently induces injury in extrahepatic organs, including the lung, the kidney and the heart (1,2). Understanding the pathophysiological process of liver reperfusion injury is clinically and pathophysiologically important.

Ischemic preconditioning, which is defined as multiple cycles of brief ischemia and reperfusion before a prolonged ischemic insult, has been reported to exert protection in several organs, resulting in increased tolerance toward organ hypoxia. Ischemic preconditioning has been shown to attenuate the tissue injury observed after reperfusion of the liver (3–5). Several mediators, including adenosine, have been shown to play a crucial role in the protective response of ischemic preconditioning (3–6).

In the present study, we focused on adenosine and its endogenous metabolic derivate, inosine, to observe their effects in an *in vitro* model of liver I-R injury. For a long time inosine was considered to be an inactive metabolite. However, several studies have shown that it has immunomodulatory, neuroprotective, cardioprotective and cytoprotective effects (7–10). These effects have been attributed to several independent mechanisms. First, inosine can bind to A_2A_ adenosine receptors activating several receptor dependent intracellular signaling pathways (11,12). Second, previous studies showed in kidney epithelial cells that inosine serves as an alternative substrate for ATP generation during hypoxia (13,14). Third, inosine (but not adenosine) can inhibit the activation of poly(ADP-ribose) polymerase enzyme (PARP) preserving cells from a suicidal utilization of NAD^+^ and ATP and, subsequently, cell death (15).

In this study, we evaluated the potential cytoprotective effects of adenosine and inosine in a cell-based model of liver I-R injury and pharmacologically characterized their mode of action.

## Materials and methods

### Materials

Adenosine, inosine, 8-cyclopentyl-1,3-dipropylxanthine (CDPX), 8-(3-chlorostyryl) caffeine (CSC), alloxazine, MRS 1523 and erythro-9-(2-hydroxy-3-nonyl) adenine hydrochloride (EHNA) were obtained from Sigma-Aldrich (St. Louis, MO, USA). 4-amino-5-(3-bromophenyl)-7-(6-morpholinopyridin-3-yl)pyrido[2,3-d]pyrimidine, 2HCl (ABT 702) was purchased from Calbiochem-Merck, Darmstadt, Germany. The receptor antagonists and ABT 702 were dissolved in dimethylsulfoxide (DMSO): dilutions were made in phosphate-buffered saline (PBS, pH 7.4) to obtain a final 0.5% DMSO content in the assay volume. EHNA was dissolved in distilled water. Adenosine and inosine were dissolved in DMEM.

The article "Adenosine and inosine exert cytoprotective effects in an in vitro model of liver ischemia-reperfusion injury" was published in 2012. Journal: Int J Mol Med.

### Cell culture

The human hepatocellular carcinoma-derived cell line HepG2 was obtained from the European Collection of Cell Cultures (Salisbury, UK) and maintained in Dulbecco’s modified Eagle’s medium (DMEM) supplemented with 4.5 g/l glucose and 10% fetal bovine serum (Invitrogen, Carlsbad, CA, USA), 4 mM glutamine, 100 IU/ml penicillin and 100 *μ*g/ml streptomycin. Five days prior to the assay 10,000 cells/well were plated into 96-well tissue culture plates and cultured at 37°C in a 5% CO_2_ atmosphere. Cells from passage numbers 9–25 were used for subsequent assays.

### In vitro liver ischemia-reperfusion model

We developed a cell-based assay of liver ischemia-reperfusion in HepG2 human liver epithelial cells. HepG2 cells were plated into 96-well tissue culture plates. Cells were cultured for 5 days to form a confluent monolayer for the following assay. Culture medium was replaced with DMEM containing no glucose (Biochrom AG, Berlin, Germany) prior to induction of hypoxia. Culture plates were placed in gas-tight incubation chambers (Billups-Rothenberg Inc., Del Mar, CA, USA) and the chamber atmosphere was replaced by flushing the chamber with 95% N_2_: 5% CO_2_ mixture at 25 l/min flow rate for 5 min. The hypoxic chamber was sealed and incubated at 37°C for various time periods. Following hypoxia, the culture medium was removed and fresh DMEM containing 4.5 g/l glucose supplemented with 10% serum was added and the cells underwent re-oxygenation at 37°C in a 5% CO_2_ atmosphere for various time periods depending on the specific experimental protocol. Cells exposed to hypoxia in complete culture medium served as controls (CTL), as no reduction was detected in cell viability compared to cells maintained in normal culture conditions (complete culture medium, 5% CO_2_ atmosphere, 37°C), if HepG2 cells were exposed to oxygen depletion with culture medium containing 4.5 g/l glucose and 10% serum for 24 h.

Inosine and adenosine proved to be markedly cytoprotective in our *in vitro* cell-based assay of liver I-R injury. In various studies we tested different periods of hypoxia (0-14-24 h) and subsequent re-oxygenation (0-4-24 h) in HepG2 cultures. Four groups were studied (n=24 for each group). The first group received pretreatment with adenosine, while the second group was pretreated with inosine prior to combined oxygen-glucose deprivation (COGD) conditions (from 300–1,000 *μ*M, applied 10 min before hypoxia). The third group (control) was subjected to COGD with drug vehicle only. The fourth group was the negative control group of the assay in which the cells were cultured in glucose containing medium (4.5 g/l) during the entire assay period. At the end of the experiments 3-(4,5-dimethyl-2-thiazolyl)-2,5-diphenyl-2H-tetrazolium bromide (MTT) viability and lactate dehydrogenase (LDH) cytotoxicity assays were conducted as described below.

The article "Adenosine and inosine exert cytoprotective effects in an in vitro model of liver ischemia-reperfusion injury" was published in 2012. Journal: Int J Mol Med.

### Pharmacological characterization of the cytoprotective effects of adenosine and inosine in the in vitro model of liver I-R

The concentration-dependence of the cytoprotective effects was tested in HepG2 cells subjected to COGD with adenosine or inosine pretreatment (1, 3, 10, 30, 100, 300, 1,000–3,000 *μ*M, n=3 each). The effects of adenosine and inosine were compared on the same 96-well tissue culture plate. A_1_ adenosine receptor antagonist CDPX (16,17), selective A_2A_ antagonist CSC (18,19), the selective A_2B_ adenosine receptor antagonist alloxazine (20), and the A_3_ adenosine receptor antagonist MRS 1523 (21,22) were added 30 min prior to adenosine or inosine (300 *μ*M) in the indicated concentration prior to COGD. The cytotoxicity of receptor antagonists was also tested under normoxic conditions.

The adenosine deaminase inhibitor EHNA (23) and the adenosine kinase inhibitor ABT 702 (24,25) were applied at 10 and 30 *μ*M prior to administering adenosine or inosine and COGD. The combined administration of EHNA and ABT 702 was also investigated. In all analyses, all relevant assay conditions (including adenosine receptor antagonists assays, adenosine and inosine comparisons) were represented on the same 96-well tissue culture plate to prevent inter-plate assay variability. The experiments were repeated independently at least three times.

### MTT cell viability assay

To estimate the number of viable cells, MTT was added to the cells at a final concentration of 0.5 mg/ml and cultured at 37°C in a 5% CO_2_ atmosphere for 1 h (26). The incubation medium was removed and the converted formazan dye was dissolved in isopropanol and measured at 570 nm with background measurement at 690 nm on a PowerWave reader (BioTek Instruments,. Inc., Winooski, VT, USA). A calibration curve was created by measuring the converting capacity of MTT of serial dilutions of HepG2 cells. The viable cell count was calculated using Gen5 data reduction software.

### LDH cytotoxicity assay

Cell culture supernatant (30 *μ*l) was mixed with 100 *μ*l freshly prepared LDH assay reagent to reach final concentrations of 85 mM lactic acid, 1040 mM nicotinamide adenine dinucleotide, 224 mM N-methylphenazonium methyl sulfate, 528 mM 2-(4-iodophenyl)-3-(4-nitrophenyl)-5-phenyl-2H-tetrazolium chloride and 200 mM Tris (pH 8.2). The changes in absorbance were read kinetically at 492 nm for 15 min. LDH activity values are shown as Vmax in mOD/min for kinetic assay (27).

The article "Adenosine and inosine exert cytoprotective effects in an in vitro model of liver ischemia-reperfusion injury" was published in 2012. Journal: Int J Mol Med.

### Statistical analysis

Data are shown as the means ± SEM. One-way ANOVA was used to detect differences between groups. Post hoc comparisons were made using Tukey’s test. A value of P<0.05 was considered to indicate statistically significant differences. All statistical calculations were performed using GraphPad Prism 5 analysis software.

## Results

### Characterization of an in vitro liver ischemia-reperfusion model in HepG2 cells

To develop a reproducible *in vitro* liver ischemia reperfusion model on HepG2 liver epithelial cells, we tested different periods (12, 14 and 24 h) of COGD, followed by a subsequent re-oxygenation period of 4 h (Fig. 1). Twelve hours of hypoxia combined with 4 h of re-oxygenation did not induce a significant decline of the cell viability (data not shown). However, 14 h of hypoxia combined with 4 h re-oxygenation induced a significant decline of the cell viability. Furthermore, 24 h of hypoxia followed by a 4 h re-oxygenation period markedly reduced cellular viability in all groups, as detected by MTT viability assay. Both 14 and 24 h of COGD were associated with a significant elevation of LDH activity detected in the cell culture supernatant (Fig. 1).

Various re-oxygenation periods (0-4-24 h) were also investigated after 14 h-long COGD. Increased cell injury was detected through the progression of the re-oxygenation period, as measured by both MTT and LDH assays (Fig. 2). Overall, these data indicate that in the current assay a substantial degree of cell injury occurs during the hypoxic period.

### Effects of adenosine and inosine in an in vitro model of liver ischemia-reperfusion

Adenosine and inosine significantly protected against the loss of cell viability of HepG2 cultures during 14 and 24 h of the COGD group, and reduced LDH release from the cells (Fig. 3). Although adenosine and inosine significantly protected HepG2 cultures from 14 h hypoxia injury, during the progression of the re-oxygenation phase a progressive reduction in cell viability and enhanced LDH enzyme release were detected in all groups, as assessed by the MTT and LDH assays. These findings are consistent with the hypothesis that an extended hypoxia results in further cell damage during the reoxygenation (reperfusion) phase. Thus our *in vitro* model clearly demonstrates the main aspects of the *in vivo* liver ischemia-reperfusion injury, with subsequent secondary injury occurring in the reperfusion phase.

The article "Adenosine and inosine exert cytoprotective effects in an in vitro model of liver ischemia-reperfusion injury" was published in 2012. Journal: Int J Mol Med.

### Pharmacological characterization of the effects of adenosine and inosine in an in vitro liver ischemia-reperfusion model

For subsequent in-depth characterization of the effects of adenosine and inosine, we selected 14 h of hypoxia and 4 h of re-oxygenation periods as the standard assay conditions. First, we established a dose-response comparison between the cytoprotective effects of adenosine and inosine, by testing each compound in a concentration range of 1 *μ*M – 3 mM. Adenosine and inosine showed cytoprotective effects already at 300 *μ*M, and reached their maximum cytoprotective effect at 1,000 *μ*M (Fig. 3). Adenosine and inosine partially attenuated cellular LDH release, starting already at the concentration of 3 *μ*M (Fig. 3).

We next evaluated the potential involvement of adenosine receptors in the protective effects of adenosine and inosine. Cells were pretreated with the adenosine receptor antagonists CDPX, CSC, alloxazine, and MRS 1523 prior to administration of cytoprotective concentrations (300 *μ*M) of adenosine or inosine. None of the adenosine receptor antagonists affected the cytoprotective effects of adenosine and inosine during COGD and following a 4 h-long re-oxygenation period (Fig. 4). These data suggest that adenosine and inosine exert their cytoprotective effects by receptor-independent pathways.

The adenosine deaminase inhibitor EHNA (10 *μ*M) almost fully reversed the protective effect of 300–1,000 *μ*M adenosine during COGD and following a 4 h-long re-oxygenation period (Fig. 5). On the other hand, EHNA did not influence the cytoprotective effect of inosine in same assay conditions (Fig. 5). The adenosine kinase inhibitor ABT 702 (30 *μ*M) significantly reversed the protective effect of 300 and 1,000 *μ*M adenosine and inosine during COGD and following a 4 h-long re-oxygenation period. We also tested both enzyme inhibitors in combined administration (Fig. 7). Notably, ABT 702, on its own, appeared to have a mild cytoprotective effect in our assay (Figs. 6 and 7).

## Discussion

The present study utilizes a cell-based model of liver ischemia-reperfusion injury in cultured HepG2 cells subjected to combined oxygen-glucose deprivation followed by re-oxygenation. Experimental conditions similar to the current ones have previously been used in multiple studies in cultured hepatocytes and Kupffer cells to mimic conditions of ischemia, in order to study pathways of cell death, signal transduction, free radical and oxidant production and inflammatory responses (28–33). Our results demonstrate that both adenosine and inosine exert cytoprotective effects in the current model, in a concentration-dependent manner (when assessed by measurement of LDH release and mitochondrial activity by the MTT assay). Although in several experimental models the cytoprotective effects of adenosine and inosine are known to be dependent on activation of adenosine A_2A_ receptors (11,12,34), the results of the current study demonstrate that the protective effect of adenosine and inosine in the current experimental conditions were not mediated by adenosine receptor-dependent pathways, as evidenced by the failure of specific adenosine receptor blockers to prevent the protective effects. Although several reports suggest a role for cell surface adenosine receptors in the reduction of liver reperfusion injury *in vivo* (35–39), it is likely that the location of these receptors is primarily on mononuclear cells involved in pro-inflammatory/immune responses (as opposed to hepatocytes).

The article "Adenosine and inosine exert cytoprotective effects in an in vitro model of liver ischemia-reperfusion injury" was published in 2012. Journal: Int J Mol Med.

While adenosine receptors failed to play a role in the cytoprotective effects of adenosine and inosine described in the present study, the data suggest the involvement of receptor-independent intracellular actions that are related to a direct regulation of cellular bioenergetics. We utilized the pharmacological inhibitor EHNA to inhibit adenosine deaminase, the enzyme that is responsible for the intracellular conversion of adenosine to inosine. EHNA significantly decreased the viability of the adenosine-treated cells subjected to COGD and also significantly increased the LDH release from the cells (Fig. 5). On the other hand, EHNA did not reduce the protective effect of inosine. These data are consistent with the hypothesis that, ultimately, an intracellular action, mediated by inosine, is responsible for the protective effect of adenosine. Our interpretation of the experimental findings is that, similar to astrocytes and kidney epithelial cells subjected to hypoxia and re-oxygenation (13,14,23), the conversion of adenosine to inosine and its subsequent metabolism to ribose-phosphate, followed by ATP generation via the pentose phosphate pathway are responsible for the observed cytoprotective effects.

Haun *et al* (23), Jurkowitz *et al* (40) and Litsky *et al* (41) demonstrated that the ribose moiety of the adenosine and inosine can be used as a precursor for phosphorylated glycolytic intermediates in reactions catalyzed by enzymes of the pentose phosphate pathway. The first reaction in this pathway is the phosphorolysis of inosine and the formation of ribose 1-phosphate or hypoxanthine, which is catalyzed by purine nucleoside phosphorylase. Three ribose 1-phosphates are isomerized to three D-ribose 5-phosphates, which then convert to two fructose 6-phosphates and one glyceraldehyde 3-phosphate, via transaldolases and transketolases of the pentose phosphate pathway. These phosphorylated intermediates enter the glycolytic pathway yielding a net production of 8 moles ATP and 5 moles NADH + H^+^ from three molecules of ribose 1-phosphate (Fig. 8). All produced NADH + H^+^ convert to NAD^+^ by lactate dehydrogenase (LDH) in anaerobic conditions. However, after a while, lactate accumulates resulting in cellular acidosis. For abolishing the acidosis lactate degradation to pyruvate and its further decomposition in the Krebs cycle at the presence of oxygen is indispensable.

The article "Adenosine and inosine exert cytoprotective effects in an in vitro model of liver ischemia-reperfusion injury" was published in 2012. Journal: Int J Mol Med.

From the same molar amount (3 moles) of extracellular (or exogenous) glucose: 6 moles of ATP and 6 moles of NADH + H^+^ are produced during the glycolysis (Fig. 8). From the breakdown of glycogen, 3 moles of intracellular glucose-1 phosphate can produce a maximum of 9 moles of net ATP and 6 moles of NADH + H^+^. On the other hand, from 3 moles of adenosine or inosine, the cell can produce net 8 moles of ATP and 5 moles of NADH + H^+^. Thus, the cells tend to elevate the intracellular NAD+/NADH + H^+^ ratio, thereby regenerating as many NADH + H^+^ molecules as possible within a short time.

On the other hand, NAD^+^ molecules are required to continue the glycolysis and lactate intermediates inhibit the further regeneration if the NADH + H^+^ molecules thereby impairing glycolysis. During excessive hypoxia, the accumulation of NADH + H^+^ occurs and, subsequently, inhibition of several enzymes (citrate synthase, isocitrate-dehydrogenase, α-ketoglutarate dehydrogenase) occurs, thereby interfering with the Krebs cycle, which is controlled by the ratio of the NADH/NAD^+^ and the ATP/ADP. Furthermore, during massive anaerobic conditions, NADH + H^+^ accumulation also leads to an inhibition of glycolysis. In summary, during COGD, adenosine and inosine may delay the accumulation of NADH + H^+^ and they can serve as a source of energy to maintain basal cellular function. In prolonged hypoxia, the accumulation of NADH + H^+^ is inevitable and the glycolysis and the Krebs cycle are both inhibited. Thus, long-term absence of the terminal oxidation and the regeneration of NADH + H^+^ to NAD^+^ result in severe cellular energy imbalance.

The results of the present study also demonstrated that the administration of the adenosine kinase inhibitor ABT 702 reversed all of the protective effects of adenosine and inosine. These findings are consistent with the hypothesis that adenosine kinase is responsible for producing AMP, ADP, and, eventually, ATP from adenosine. When sufficient ADP molecules are present in the cells, ATP can be created from ADP both via the adenosine kinase-mediated route and via the pentose phosphate pathway. The inhibition of the adenosine kinase pathway by ABT 702 results in less ADP production in the adenosine kinase-mediated pathway, which induces less ATP generation in the pentose phosphate shunt as well. This mechanism explains that, i) ATP production of the pentose phosphate pathway depends on the amount of ADP molecules derived from the adenosine kinase mediated route, and ii) provides evidence that administration of adenosine kinase inhibitor ABT 702 reversed all of the protective effects of adenosine and inosine. Furthermore, adenosine kinase inhibitor (ABT 702) administration without exogenous adenosine or inosine affords a mild cytoprotective effect, but prevents the cytoprotection provided by exogenous adenosine or inosine (Figs. 6 and 7).

The article "Adenosine and inosine exert cytoprotective effects in an in vitro model of liver ischemia-reperfusion injury" was published in 2012. Journal: Int J Mol Med.

Our data and the above considerations, taken together, indicate that adenosine and inosine may exert some of their cytoprotective effects under our current experimental conditions by stepping in as an emergency energy source, when glucose is insufficient to support cellular functions. This hypothesis is supported both by several reports in the literature where cellular ATP levels were elevated in ischemic or hypoxic cells treated with adenosine or inosine (23,40,42–44) as well as by our measurements (13,14). Although we have not directly measured the transport of adenosine or inosine into the cells, previous studies have demonstrated that these purines can readily enter the cells (23,40). We propose that the two processes, i) degradation of adenosine and inosine via the pentose-phosphate pathway, and ii) the phosphorylation of adenosine to AMP, are required in a well-balanced parallel fashion. Our hypothesis is that both pathways are necessary at the same time to support the generation of ATP under hypoxic conditions. The first process provides the energy, while the second one supplies the substrate (e.g. adenosine, AMP, ADP) to convert it into a high energy intermediate that conserves it in a ready-to-use form. Markedly, the combined blockage of adenosine deaminase (by EHNA) and adenosine kinase (by ABT 702) resulted in no further reduction in cell viability after COGD (as compared to either inhibitor), which supports that these enzymes take part in the same cytoprotective mechanism (Fig. 7).

In conclusion, it is likely that the cytoprotective effects of adenosine and inosine involve multiple, parallel and interrelated mechanisms under the current experimental conditions. During ischemia and inflammation, the concentration of purine metabolites increases dramatically in the extracellular space. ATP degrades into AMP and subsequently to adenosine, which may be released from the cells and appears in the extra-cellular space. Inosine can be formed from adenosine with an adenosine deaminase enzyme, which occurs both intra- and extracellularly. Consistent with these notions, there are several reports that demonstrate the cytoprotective effect of endogenously formed adenosine in the context of acute ischemic injury of the liver (45,46).

The article "Adenosine and inosine exert cytoprotective effects in an in vitro model of liver ischemia-reperfusion injury" was published in 2012. Journal: Int J Mol Med.

The current study shows that adenosine and inosine are cytoprotective on HepG2 cultures exposed to combined oxygen-glucose deprivation. This protective effect is not mediated by a receptor-dependent pathway, but it is likely mediated by maintenance of cellular bioenergetics due to the utilization of adenosine and inosine as alternative substrates for ATP generation.

While the therapeutic utilization of adenosine as a hepatoprotective agent *in vivo* is difficult due to its short half-life and adverse cardiovascular side-effect profile, inosine may emerge as a potential candidate. Indeed, several recent studies have demonstrated that administration of inosine can be protective against various forms of ischemic conditions (7–10). The current results may provide a mechanistic explanation to the previously reported protective effect of inosine *in vitro* as an adjuvant to organ storage solutions (47) or *in vivo* as a protective agent in a rat model of hepatic reperfusion injury (48) and can stimulate further studies to explore whether inosine has the potential to improve cellular bioenergetics and to protect hepatocytes in various forms of liver injury, including various forms of warm ischemia or cold ischemia associated with liver transplantation.

## Figures and Tables

**Figure 1.** Viability and LDH activity are shown in HepG2 cultures during different periods of combined oxygen-glucose deprivation (COGD) and following a 4 h-long re-oxygenation. (A) Percent viability values by MTT assay and (B) LDH activities in mOD/min are shown. Each group, except the control (CTL) group, was incubated in glucose-free medium under anaerobic conditions for 14- or 24-h periods and a subsequent 4 h-long re-oxygenation phase by normalizing glucose and oxygen levels in the cell culture medium and atmosphere. Data are shown as the means ± SEM (n=24 for each group). White bar is control (CTL) group, black bar is COGD group during COGD without any pharmacological pretreatment, dotted bar shows 300 *μ*M adenosine (ADE) pretreatment group and ruled bar represents 300 *μ*M inosine (INO) pretreatment group. ADE and INO groups were also under COGD conditions. ^#^P<0.05 compared to the CTL group and ^*^P<0.05 compared to the COGD group.

The article "Adenosine and inosine exert cytoprotective effects in an in vitro model of liver ischemia-reperfusion injury" was published in 2012. Journal: Int J Mol Med.

**Figure 2.** Viability and LDH activity are shown in HepG2 cultures during a 14 h-long combined oxygen-glucose deprivation (COGD) and following 0-4-24 h of re-oxygenation. (A) Percent viability values by MTT and (B) LDH activities in mOD/min are shown. Each group, except the control (CTL) group, was incubated in glucose-free medium under anaerobic conditions for a 14 h-long period and following a 0-4-24 h-long re-oxygenation phase by normalizing glucose and oxygen levels in the cell culture medium and atmosphere. Data are shown as the means ± SEM (n=24 for each group). White bar is control (CTL) group, black bar is COGD group during COGD without any pharmacological pretreatment, dotted bar shows 300 *μ*M adenosine (ADE) pretreatment group and ruled bar represents inosine pre-treatment group at 300 *μ*M (INO). ADE and INO groups were also under COGD conditions. ^#^P<0.05 compared to the CTL group and ^*^P<0.05 compared to the COGD group.

**Figure 3.** Dose-response effects of (A and B) adenosine and (C and D) inosine on percent viability values by MTT assay and LDH activities in mOD/min in HepG2 cultures exposed to a 14 h-long combined oxygen-glucose deprivation (COGD) and a subsequent 4 h-long re-oxygenation. Each group, except the control (CTL) group, was incubated in glucose-free medium under anaerobic conditions for a 14 h-long period and following a 4 h-long re-oxygenation phase by normalized glucose and oxygen levels in the cell culture medium and atmosphere. Data are shown as the means ± SEM. White bar is control (CTL, n=16) group in the control conditions of the assay, black bar is COGD group (n=32) during COGD without any pharmacological pretreatment, dotted bar shows the adenosine pretreatment group at 1, 3, 10, 30, 100, 300, 1,000 and 3,000 *μ*M (ADE) and ruled bar represents the inosine pretreatment group at 1, 3, 10, 30, 100, 300, 1,000 and 3,000 *μ*M (INO). ADE and INO groups (n=3) were also under COGD conditions. ^#^P<0.05 compared to the CTL group and ^*^P<0.05 compared to the COGD group.

**Figure 4.** Effect of adenosine receptor antagonists on the cytoprotective effects of inosine. Confluent HepG2 cultures were subjected to combined oxygen-glucose deprivation (COGD, n=32) for 14 h followed by a 4-h-long re-oxygenation period. (A and B) The A_1_ adenosine receptor antagonist, CDPX, (C and D) the A_2A_ adenosine receptor antagonist, CSC, (E and F) the A_2B_ adenosine receptor antagonist, alloxazine, and the A_3_ adenosine receptor antagonist, (G and H) MRS 1523 were applied in the indicated concentrations (n=3) 30 min prior to the inosine or adenosine pretreatment (INO or ADE, n=12) and were present throughout the COGD period. Viability was measured by the MTT assay (A, C, E and G) and LDH activities (B, D, F and H) were measured from the cell culture supernatant. Controls (CTL, n=16) were exposed to hypoxia in complete culture medium. Data are shown as the means ± SEM. ^#^P<0.05 compared to CTL and ^*^P<0.05 compared to COGD. None of the adenosine receptor antagonists affected the cytoprotective effects of adenosine (data not shown) and inosine during COGD.

The article "Adenosine and inosine exert cytoprotective effects in an in vitro model of liver ischemia-reperfusion injury" was published in 2012. Journal: Int J Mol Med.

**Figure 5.** Effect of adenosine deaminase inhibitor (EHNA) on the cytoprotective action of 300–1,000 *μ*M adenosine (ADE) and inosine (INO) in HepG2 cultures exposed to a 14 h-long hypoxia period and a subsequent 4 h re-oxygenation. Data are shown as the means ± SEM. (A and C) Percent viability values by MTT assay and (B and D) LDH activities in mOD/min are shown. Seven groups were studied both of the adenosine and inosine. The COGD group during COGD (black bar, n=16), a COGD group plus 10 *μ*M EHNA during COGD (black bar, n=16), groups pre-treated with 300 or 1,000 *μ*M adenosine (ADE) and inosine (INO) during COGD (ADE, dotted bar; INO, ruled bar, n=3) and finally groups pre-treated with 300 or 1,000 *μ*M adenosine and inosine plus 10 *μ*M EHNA during COGD (ADE 300–1,000 *μ*M + EHNA and INO 300–1,000 *μ*M + EHNA are grey bar, n=3). The white bar is the control (CTL, n=16) group and represents the negative control of the assay. ^#^P<0.05 compared to CTL; ^*^P<0.05 compared to the COGD group; and ^δ^P<0.05 compared to the 300–1,000 *μ*M ADE groups.

**Figure 6.** Effect of adenosine kinase inhibitor (ABT 702) on the cytoprotective action of 300–1,000 *μ*M adenosine (ADE) and inosine (INO) in HepG2 cultures exposed to a 14 h-long hypoxia period and a subsequent 4 h re-oxygenation. Data are shown as the means ± SEM. (A and C) Percent viability values by MTT assay and (B and D) LDH activities in mOD/min are shown. Seven groups were studied both of the adenosine and inosine. The COGD group during COGD (black bar, n=16), a COGD group plus 30 *μ*M ABT 702 during COGD (black bar, n=16), groups pre-treated with 300 or 1,000 *μ*M adenosine (ADE) and inosine (INO) during COGD (ADE, dotted bar; INO, ruled bar, n=3) and finally groups pre-treated with 300 or 1,000 *μ*M adenosine and inosine plus 30 *μ*M ABT 702 during COGD (ADE 300–1,000 *μ*M + ABT and INO 300–1,000 *μ*M + ABT are grey bars, n=3). The white bar is the control (CTL, n=16) group and represents the negative control of the assay. ^#^P<0.05 compared to CTL; ^*^P<0.05 compared to the COGD group; and ^δ^P<0.05 compared to the 300–1,000 *μ*M ADE and INO groups.

**Figure 7.** Collective effect of adenosine deaminase inhibitor (EHNA) and adenosine kinase inhibitor (ABT 702) on the cytoprotective actions of 300–1,000 *μ*M adenosine (ADE) and inosine (INO) in HepG2 cultures exposed to a 14 h-long hypoxia period and a subsequent 4 h re-oxygenation. Data are shown as the means ± SEM. (A and C) Percent viability values by MTT assay and (B and D) LDH activities in mOD/min are shown. Seven groups were studied both of the adenosine and inosine. The COGD group during COGD (black bar, n=32), a COGD group plus 30 *μ*M ABT 702 during COGD (black bar, n=3), a COGD group plus 10 *μ*M EHNA during COGD (black bar, n=3), a COGD group plus 30 *μ*M ABT 702 and 10 *μ*M EHNA in combination during COGD (black bar, n=3), groups pre-treated with 300–1,000 *μ*M adenosine (ADE) and inosine (INO) during COGD (ADE, dotted bar; INO, ruled bar, n=3) and finally groups pre-treated with 300 or 1,000 *μ*M adenosine and inosine plus 30 *μ*M ABT 702 or 10 *μ*M EHNA during COGD (ADE/INO 300/1,000 *μ*M + ABT 702/EHNA or in combination are grey bars, n=3). The white bar is the control (CTL, n=16) group and represents the negative control of the assay, subjected to hypoxia in complete culture medium. ^#^P<0.05 compared to CTL; ^*^P<0.05 compared to the COGD group; and ^δ^P<0.05 compared to the 300–1,000 *μ*M ADE and INO groups.

The article "Adenosine and inosine exert cytoprotective effects in an in vitro model of liver ischemia-reperfusion injury" was published in 2012. Journal: Int J Mol Med.

**Figure 8.** Scheme representing some of the proposed metabolic pathways for the conversion of adenosine and inosine into different substrates for the glycolytic pathway. The diagram also shows an alternative way to produce energy in the absence of glucose during hypoxic injury.

## Abbreviations:

ABT 702: 4-amino-5-(3-bromophenyl)-7-(6-morpholino-pyridin-3-yl)pyrido[2,3-d]pyrimidine, 2HCl;
CDPX: 8-cyclopentyl-1,3-dipropylxanthine;
CSC: 8-(3-chlorostyryl) caffeine;
COGD: combined oxygen-glucose deprivation;
DMEM: Dulbecco’s modified Eagle’s medium;
DMSO: dimethylsulfoxide;
EHNA: erythro-9-(2-hydroxy-3-nonyl) adenine hydrochloride;
I-R injury: ischemia-reperfusion injury;
LDH: lactate dehydrogenase;
MTT: 3-(4,5-dimethyl-2-thiazolyl)-2,5-diphenyl-2H-tetrazolium bromide;
PBS: phosphate-buffered saline.
